The article "Complementary and Integrative Approaches to Cancer: A Pilot Survey of Attitudes and Habits among Cancer Patients in Italy" was published in 2022. Journal: Evid Based Complement Alternat Med.

# Complementary and Integrative Approaches to Cancer: A Pilot Survey of Attitudes and Habits among Cancer Patients in Italy

**DOI:** 10.1155/2022/2923967

**Published:** 2022-08-01

**Authors:** Massimo Bonucci, Andrea Geraci, Dina Pero, Cristina Villivà, Daniele Cordella, Maria Condello, Stefania Meschini, Laura del Campo, Franco Tomassi, Alessandro Porcu, Francesco De Lorenzo, Francesco Lozupone

**Affiliations:** ^1^Association for Research on Integrative Oncological Therapies (ARTOI), Roma, Italy; ^2^Italian Center for Global Health, Istituto Superiore di Sanità, Roma, Italy; ^3^Italian Association for Cancer Patients, Relatives and Friends (AIMaC), Roma, Italy; ^4^Directorate-General Information Technology Unit, Istituto Superiore di Sanità, Roma, Italy; ^5^National Center for Drug Research and Evaluation, Istituto Superiore di Sanità, Roma, Italy

## Abstract

**Background:**

Cancer patients are among the main consumers of traditional, complementary, integrative, and alternative medicine (TCIM) such as natural products (herbals, integrators, etc.) and mind and body practices (yoga, acupuncture, etc.).

**Methods:**

A questionnaire on TCIM was submitted to 415 Italian cancer patients. The questionnaire consisted of three sections: (i) biographical and clinical information; (ii) use of natural substances; and (iii) use of mind-body practices.

**Results:**

406 patients completed the questionnaire. The prevalence of TCIM use was 72.3%. Of them, 75.6% started to use TCIM after a tumor diagnosis. The main reasons for using TCIM were to mitigate side effects (65.0%), to regain physical and mental balance (35.9%), to relieve pain (18.3%), and to improve the efficacy of cancer therapy (16.0%). 44.7% of patients taking natural products used them during conventional therapies (chemotherapy, radiotherapy, etc.), and in 67.5% of cases without consulting a doctor. As a consequence, only about 50% of patients taking natural substances used these compounds appropriately, and the most common errors were related with the purpose of reducing the side effects of the therapy (52.3%) and for boosting immune system (32.1%).

**Conclusions:**

There is an impelling need to provide patients with scientifically validated information to raise awareness about the benefits and risks of using TCIM.

## 1. Introduction

According to the International Agency of Research on Cancer (IARC), 1 in 5 people in the world will develop cancer in their lifetime, and about 8% women and 12% men die from this pathology. Breast cancer is the most commonly diagnosed cancer (6.9%), and together with lung cancer it remains the leading cause of cancer death, with an estimated 1.8 million deaths (18%), followed by colorectal (9.4%), liver (8.3%), and stomach (7.7%) [1]. Although in the last years early detection and effective treatments have reduced mortality rates, they remain high, particularly in low-income countries [2, 3]. Moreover, cancer therapies are often accompanied by severe side effects that not only affect the quality of life, but can also lead to more suffering and to a reduced response to treatments [4, 5]. This is why an increasing number of patients is turning to unconventional approaches, i.e., complementary medicines, hoping to improve the outcomes [6–9].

The World Health Organization (WHO) defines complementary medicine as “a set of health practices that are not part of a country's tradition or conventional medicine and are not fully integrated into the dominant health system.” In 2017, the WHO unit of traditional and complementary medicine (TCM) unit was redefined to include the term “integrative medicine”, in order to increase the integrative approaches of both TCM and conventional medicine and in relation to social policy, as well as to knowledge and practice. The unit is now officially named “traditional, complementary, and integrative medicine (TCIM)” [10]. The US National Center for Complementary and Integrative Health (NCCIH) divides complementary and alternative medicine into the following: (i) biological products (BP), including vitamins and minerals, herbal, and probiotics products; (ii) mind-body practices (MBP), such as yoga, meditation, qigong, acupuncture, and spinal manipulation (both chiropractic and osteopathic), relaxation, hypnotherapy, and Pilates; and (iii) other complementary health approaches that may not fit neatly into any of these groups, such as traditional healing practices, Ayurvedic medicine, traditional Chinese medicine, homeopathy, and naturopathy [11].

Recently, an increasing number of publications show the beneficial anticancer effects of traditional or newly discovered herbals and their active metabolites, with some of them also able to overcome multidrug resistance and minimize harmful side effects caused by radiotherapy and chemotherapy [12–18].

Despite the growing interest of healthcare professionals in TCIM and the increasing number of scientifically validated studies, patients often turn to TCIM without professional input, taking information from unverifiable sources such as social networks, friends, and other patients, taking these products as self-medication [19–21], often underestimating the risks of adverse events, especially when taken in combination with chemotherapy (CT) [22–25]. Patients expect as main benefits a reduction of chemotherapy side effects, damage avoidance or minimization, boosting the immune system, and improvement of the response to conventional therapies [26, 27].

This study aims to assess the prevalence of TCIM among cancer patients in Italy. Our goal was to analyze the use of TCIM during conventional therapies, paying particular attention to those patients who declared to take TCIM as self-medication, in order to highlight the risks of TCIM use in combination with conventional drugs. The novelty of this work lies in the fact that the information was collected exclusively from the patients and not from healthcare professionals, who were often unaware. The oncological characteristics, the TCIM methods chosen, at what stage of therapy they were taken, and the frequency of use were also examined. In addition, we assessed the source of information, patients' expectations towards these compounds, and if their expectations were fulfilled.

## 2. Methods

### 2.1. Data Sources and Patients Setting

A descriptive cross-sectional survey was conducted between April 2018 and May 2019 to collect data on cancer patients' choices of TCIM. Patients were asked to complete the questionnaire using the online form, available on the web portals of the Italian Institute of Health, AIMaC and ARTOI websites, or the paper form, offered to patients at the AIMaC and ARTOI information points, located in the main oncologic hospitals and in the waiting rooms of the oncologists who kindly participated in the project. All papers and electronic questionnaires collected were returned to the investigators and then the data were coded for analysis, in compliance with EU Regulation 2016/679 established by the European Parliament and Council on April 27, 2016 for the protection of individuals, with particular regard to the processing of personal data and the free movement of such data. Patients completed the questionnaire anonymously, and without assistance.

Patients' participation was on a voluntary basis and did not interfere with their medical treatment. All participating patients received information about the study. Patients were considered eligible if they met the following inclusion criteria: they were Italian-speaking over 18 years of age, without distinction of gender, diagnosed with cancer, aware of their diagnosis, able to understand the questions, and free from any condition that made filling out the questionnaire inappropriate or burdensome for the patients themselves. This survey was approved by the Ethics Committee of the Italian National Institute of Health.

### 2.2. The Questionnaire

The questionnaire used for the survey consists of three sections: the first section concerns personal and clinical information, including demographic (age and sex) and clinical data (location of primary tumor, time since diagnosis, position in the cancer treatment pathway, and drugs received); the second section concerns the use of biological products (BP) such as vitamins and minerals, herbal and probiotics products etc., which of them was used, when they were taken (before, during, or after therapy), for how long, how often and for what purpose, who suggested them, whether or not the choice was discussed with an oncologist or health specialists and, finally, whether they had any benefit; the third section concerns MBP and follows the same criteria as the previous one. Some products that may also be routinely prescribed medical therapies, such as iron, vitamin D, and calcium supplements, were included in the BP analysis. The online questionnaire was developed using “in-house” software developed by Daniele Cordella as the SurveyPro module of the Open Source Moodle application (https://www.moodle.org) available from (https://github.com/moodle/moodle). It can be downloaded freely from GitHub at https://github.com/kordan/moodle-mod_surveypro.

### 2.3. Data Analysis

The median, range, and relative frequencies were used in the descriptive analysis. Frequency analyses and cross tables with *χ*2 tests were performed. Only the questionnaires for which at least the first section was completed were analyzed. A cut-off value of *p* < 0.05 was used. No differences were observed between data collected using online or paper questionnaires.

## 3. Results

### 3.1. Patients' Characteristics

415 patients agreed to participate in this survey. Only questionnaires in which at least the first section was completed were considered analyzable, therefore, we then evaluated the responses of 406 of the 415 patients. 76.8% of patients were women, with a median age of 56 (range 24–84), 23.2% were men with a median age of 62 years (20–93). The most frequent site of primary tumor was the breast (47.8%), followed by gastrointestinal cancers (12.3%), hematological cancers (5.7%), hepato-pancreatic-biliary tumors (5.7%), and cervical and lung tumors (3.9% each) (Figure 1).

Out of 406 patients that completed the questionnaire, 116 patients (28.6%) reported not using TCIM, 228 (56.2%) used BP, 192 (47.0%) used MBP, and 30.3% used both. Patient's therapy phases (before, during, and after therapy) and therapy categories (neoadjuvant, adjuvant, and exclusive) are shown in Table 1.

### 3.2. Analysis of Patients' Responses about TCIM Choices

As detailed in Table 2, the BP most commonly reported by patients were salts and micronutrients (40.8%), vitamins (36.0%), turmeric and curcumin-based products (35.1%), aloe extracts 13.6%, mushrooms from traditional Chinese medicine (12.7%), homeopathic products (9.6%), probiotic and polydatin (8.8%), indole-3-carbinol, and sulforaphane (7.0%). 17% of patients were taking various commercially available compounds. The most commonly used MBP were “massages and manual care” (63.4% of patients), with psychic and spiritual treatments (meditation, music and art therapy, mindfulness, etc.) 33.5%, yoga (23.6%), acupuncture (20.4%), osteopathic medicine (15.2%), reiki (14.1%), Qi gong/Tai Chi (12.6%), light sports practices, (6.8%), etc. 80.7% of patients taking BP reported taking more than one product, while more than one MBP was chosen by 41.9% patients using MBP.

When and why did patients try TCIM approaches? As shown in Table 3, more than 70% of the patients who responded to the questionnaire stated that started using TCIM immediately after diagnosis (71.1% and 79.1% for BP and MBP, respectively), and almost half of them were taking TCIM during conventional therapy (44.3% and 31.4% for BP and MBP users, respectively). Although no statistically significant differences were noted between BP and MBP users before diagnosis and therapy (not shown), the number of patients using MBP was significantly lower than that of BP patients (31.4% vs. 44.3%, *p* < 0.01). Such differences increased significantly after therapy (37.2% vs. 20.6% of patients taking BP, *p* < 0.01). Overall, 71.9% of patients reported a regular BP use, while it was slightly higher, but not statistically significant, the percentage of patients who stated to practice habitually MBP (75.9%, *p* 0.829448) (Figure 2).

The most common motivations for the use of BP were (multiple responses were allowed): improving the immune system (66.2%), mitigating side effects (44.7%), and improving the impact of cancer therapy (26.3%) (Figure 3, black bars). Regarding the choice to use MBP, the main reason was the need to regain physical and mental balance (75.9%), followed by mitigating the side effects of conventional therapy (27.2%) and relieving pain (17.3%) (Figure 3, grey bars). No significant differences were observed between the responses of women and men.

As for the process that led patients to choose the BP or MBP approaches, in our study 11.0% of BP patients and 28.3% of MBP patients made their choice on their own without consulting anyone. To these, it should be added the percentage of those who obtained information from social media or magazines (9.2 and 6.8 for BP and MBP patients, respectively), relatives, friends (24.0% and 20.9% for BP and MBP patients, respectively). However, among those taking BP, the oncologist was the main consultant (32.0%), followed by the family doctor (12.7%) and by the dietician/nutritionist (11.0%) (Table 4 left columns). In addition, 22.3% of patients who learned from unverifiable sources, did not inform their oncologist or family doctor, and 39.2% of them reported to take BP during therapy.

As regards to patients using MBP, the sources of information were healthcare professionals (29.4%), personal decision (28.3%), relative or friends (20.9%), patients' associations (11.5%), other patients (6.8%), etc. (Table 4 right columns).

Afterwards, when asked if they perceived any benefit, 90.6% of patients who made use of MBP answered in the affirmative (Figure 4(a)), while this percentage decreased significantly among patients who took BP (48.2%), and 33.3% of them did not answer (Figure 4(b)).

Finally, we compared the patients' responses on why they had taken one or more BP with the actual properties and toxicokinetic characteristics of the same products accepted by the competent body or in the scientific literature (preclinical and clinical evidences). As shown in Table 5, less than half of the BP taking patients used these compounds appropriately. 25.5% of patients chose BP for purposes not related to the actual features of the product taken, and a further 25.9% of patients took more than one product, but only some of them were correctly taken. The most common errors were found in the use of supplements to reduce the side effects of therapy (52.3%), to support the immune system (32.1%), to reinforce conventional therapies (37.3%), and 8 out of 11 patients who used BP to reduce pain used products that do not possess these properties (Table 6).

## 4. Discussion

Traditional complementary and integrative medicines are an important health resource, often underestimated, but considered by an increasing number of patients. In this study, we started a survey about the use of TCIMs by cancer patients with the aim of (i) assessing the use of these products in relation to disease stage and suggested therapies and (ii) analyzing how BP or MBP were chosen in relation to cancer therapies, to highlight the potential risks from harmful combinations.

As previously reported [8, 28–30], the BP mentioned most frequently used products by patients were herbals, accounting for almost 40% of the products, followed by vitamins, salts, and minerals. The most commonly used herbals were curcumin and aloe products, both of which were among the best-known herbal remedies with healing or soothing properties. Among MBPs, massage and manual care appear to be the most commonly used practices (63.4%), followed by mind and body practices (33.5%), yoga (23.6%), and acupuncture (20.4%) (Table 2).

An essential aspect that emerges from this survey is that patients begin to turn their attention to BP after a cancer diagnosis (more than 80% of interviewed patients), as already highlighted in several articles [6, 9, 31–35]. More importantly, nearly half of the patients said that they started taking BP while they were in therapy. In general, BP use seems to be more common among patients at an early stage of the disease (0–1 years after diagnosis), (36.0% and 21.6% for BP and MBP using patients, respectively). In contrast MBPs were more common among patients in follow-up and long-term survivors (47.9% vs. 30.7% of BP), suggesting that their choice might be related to a different way of viewing life after the cancer experience, or after the acute phase of their disease.

The main reasons of BP choices were to support the immune system (66.2%), which is often severely compromised by chemotherapy, and to reduce the side effects of chemotherapy (44.7%). As for the MBP, the main reasons were the search for psycho-health balance (75.9% of patients), understandably destabilized by the disease, to counteract the toxic effects of chemotherapy (27.2%) and to relieve pain (17.3%). In general, it can be deduced that the reasons for the complementary choices lie in the desire to achieve holistic well-being, and to optimize the therapeutic effect of conventional therapy, which can also be severely compromised by dramatic side effects, such as cachexia and chronic inflammation induced by chemotherapy, which itself can lead to severe morbidity and to a significantly increased mortality [4, 36, 37].

Another important issue that we tried to address was the source of information and how TCIM choices were discussed with the family doctor or the oncologist. As described in similar studies, more than half of the patients (53.9% of BP and 73.4% of MBP users) learned about TCIM from uncontrollable or nonprofessional sources, which cannot always guarantee correct information. In addition, approximately one third of the patients interviewed did not inform the oncologist or family doctor about the products they were taking [14, 38]. The issue of self-selected products should not be undervalued, herbal remedies in special way, are considered natural, and erroneously safe, underestimating the effects of drug/BP interactions that can seriously compromise the efficacy of the therapy or increase its toxicity [20, 39, 40]. To this end, patients' responses on their motivation to take a specific BP were compared with the actual properties and toxicological characteristics of the same product (according to scientific literature and or official reports from institutional sites). Our analysis suggested that almost half of the BPs taking patients used BPs improperly, as detailed in Table 5, 25.9% of patients chose BPs for purposes not attributable to the product they were taking, and 25.9% of patients took more than one product, but only some of them were correctly chosen. The most common errors were related to the hope of increasing chemotherapy efficacy and reducing side effects, particularly those related to a weakened immune system (Table 6).

To highlight the importance of correct information and the risks that patients run with the use of BPs, we would like to illustrate two examples taken from the questionnaire.

A 48-year-old breast cancer patient said that during the therapy with letrozole and triptorelin, an effective therapy for most hormone-sensitive cancers [41], she had taken mistletoe and nux-vomica of her own accord, to increase the effectiveness of the therapy. As well known, letrozole is metabolized by the CYP450 CYP3A4 and CYP2A6 isoenzymes. Although mistletoe appears to be effective in improving the quality of life of breast cancer patients during chemotherapy and follow-up [42, 43], the fact that raw mistletoe contains toxic constituents cannot be overlooked; moreover, high doses of mistletoe have been shown in vitro to inhibit CYP3A4 activity. Consequently, mistletoe could positively affect the metabolism of letrozole by increasing the bioavailability of the drug, but also have a negative effect by increasing the adverse effects of the drug itself [44–47]. Nux-vomica extracts are usually used in the traditional Chinese medicine for their effects on the nervous system analgesic and anti-inflammatory activity. Preclinical studies also suggest an anticancer effect in breast cancer cells; unfortunately, at high doses it can be toxic due to poisonous compounds present in its composition such as strychnine, brucine, and loganine [48, 49]. Furthermore, Nux-vomica extracts may act as inhibitors of CYP2C, CYP3A, and CYP1A2 enzymatic activity [50, 51].

The second example is a 47-year-old woman with metastatic breast cancer. In the questionnaire, she stated that she was taking AHCC (active hexose correlated compound), a shiitake mushroom extract, which the patient used to alleviate the side effects of paclitaxel and bevacizumab. The antioxidant and immunostimulant properties of AHCC have been recently described, and the use of AHCC appears to be protective against the side effects of chemotherapy. In addition, AHCC is also a potential inducer of aromatase, a key enzyme of hormone-sensitive breast cancer growth [52–54]. Finally, in patients showing the variant V158M genotype of COMT (catechol-o-methyltransferase, estrogens inactivating enzyme involved in their metabolism), AHCC reduces the effects of aromatase inhibitors as in the case of the use of letrozole [55].

## 5. Conclusions

According to the scientific literature, the results of our study have confirmed that cancer patients increasingly turn to TCIM treatments after the diagnosis with the aim to reduce symptoms and also the negative effects of anticancer treatments, with the hope of obtaining an improvement in the quality of life. However, the survey has highlighted a frequent lack of correspondence between the benefits expected by patients from specific treatments and their actual, evidence-based properties, emphasizing the potential risks coming from TCIM use without consulting healthcare providers, particularly if taken during conventional therapy. The importance of this survey is to point out the impelling need to provide reliable and scientifically validated information on the use of TCIM, not only on their biological and pharmacological properties and on their potential benefits, but also on the risks of an incorrect association with anticancer drugs. The importance of this information also has economic implications, considering the economic burden for public health systems to diagnose and treat this pathology. It is therefore understandable that a therapy that is not optimized for a patient, because it includes ancillary substances that may have conflicting effects, may also result in economic harm to the patient and to the health care economy.

## Figures and Tables

**Figure 1:** The distribution of patients by tumor type.

**Figure 2:** Frequency of use of TCIM. Frequency of use of BPs or MBP among users of BP (a) or MBP (b), respectively.

**Figure 3:** Patients' motivations for using TCIM among BP users (black bars) or MBP users (grey bars). Multiple responses were allowed.

**Figure 4:** Personal experience with TCIMs. Rate of patients and perception of benefits by patients taking BP (a)and patients taking MBP (b).

**Table 1:** TCIM and therapy phases of patients.

			BP				MBP							Both			No. of TCIM taking patients				
**A**	Distribution of TCIM users (*n* = 296 72.9%)		*n*		%		*n*			%				*n*	%		*n*			%	
			228		56.2		191			47.0%				123	30%		116			28.6%	

Therapy phase			*n*	%	*n*	%	*n*	%		*n*		%		*n*	%		*n*	%		*n*	%

**B**	*Before therapy*	Total	22		9.6%		11			5.8%				5	4.1%		20				17.2%
		Waiting for the therapy		0.0%	12	54.5%				4		36.4%								11	55.0%
		I was excised/I will undergo surgery		0.0%	10	45.5%				7		63.6%								9	45.0%
	*In therapy*	Total	104			45.6%	62					32.5%		49	39.8%		52		44.8%		
		Neoadjuvant			17	16.35%				6	9.7%									11	21.2%
		Adjuvant therapy			57	54.8%				42	67.7%									29	55.8%
		Exclusive therapy			21	20.2%				9	14.5%									10	19.2%
		Not specified			9	8.7%				5	8.1%									2	3.8%
	*After the therapy*	Total	75	32.9%			92		48.2%					50		40.7%	31			26.7%	
		Follow-up long-term survivor		0.0%	53	70.7%				52			56.5%							23	74.2%
				0.0%	22	29.3%				40			43.5%							8	25.8%
	Palliative therapy and pain management			6	22.2%		7			3.7%				3		2.4%	6			5.2%	
	Refused the therapy			5	23.8%		5			2.1%				4		3.3%	1			0.1%	
	Not specified or not known			16	7.0%		15			7.9%				12		9.8%	6			5.2%	

(**A**) Distribution of BP patients, MBP patients, or patients using both approaches, (left columns), compared to patients not taking TCIM (right columns). (**B**) Patients taking TCIM in relation to stage of therapy. TCIM : Traditional Complementary Integrative Medicine; BP, herbals integrators nutraceuticals, food supplements, etc.; MBP: mind-body practices.

**Table 2:** Rate of use of TCIM methods.

Natural products (BP)*n*=228	%	*n*	Mind and body practices (MBP) *n*=194	%	*n*
Salts, microelements, and micronutrients	40.8	93	Massages and manual healing	63.4	121
Vitamins	36.0	82	Psychic and spiritual therapies (meditation, music and art therapy, mindfulness, etc.	33.5	64
Curcumin and turmeric-based products	35.1	80	Yoga	23.6	45
Aloe extracts	13.6	31	Acupuncture	20.4	39
Mushrooms (Reiki, cordyceps, Turkey tail, Lion's mane, etc.)	12.7	29	Osteopathy	15.2	29
Homeopathic products	9.6	22	Reiki	14.1	27
Probiotics and milk enzymes	8.8	20	Qi Gong/Tai Chi	12.6	24
Polydatin	8.8	20	Light sport practices	6.8	13
Indole-3-carbinol	7.0	16	Physiotherapy	2.1	4
Sulforaphane	7.0	16			
Melatonin	6.6	15			
Omega3	4.4	10			
Artemisinin and artemisinin extracts	3.5	8			
Milk thistle	3.1	7			
Fermented papaya	3.1	7			
Boswellia serrata	2.6	6			
Astragalus	2.6	6			
More than one BP	80.7	184			
Mixtures	17.5	40	More than one MBP	41.9	80
Others or no answer	0.9	2	Others or no answer	1.6	3

% of patients taking BP (left column) or MBP (right column) as listed by patients in the questionnaire.

**Table 3:** Distribution of TCIM users in relation to diagnosis.

TCIM intake period	BP (*n*=228)				MBP (*n*=191)			
	*n*		%	%	*n*	%	*n*	%
Before diagnosis	15	6.6%			10			
After diagnosis	162	71.1%				151	5.2%	
After diagnosis, before therapy or surgery During therapy After therapy			36 101 63	15.8 44.3 27.6			22 60 86	11.5% 31.4% 45.0%
Regardless of the disease, others, or no answer	47	20.6%			71	37.2%		
	18	7.9%			14	7.3%		

**Table 4:** Sources of information on TCIM.

TCIM: sources of information	BP		MBP	
	*n*	%	*n*	%
None	25	11.0	54	28.3
Relatives or friends	55	24.1	40	20.9
Other patients	15	6.6	13	6.8
Patients' associations	7	3.1	22	11.5
Social media or magazines	21	9.2	13	6.8
Oncologists	73	32.0	32	16.8
Family doctors	29	12.7	11	5.8
Dieticians/nutritionists	25	11.0	5	2.6
Homeopathic doctors	6	2.6	1	0.5
Other physicians	7	3.1	0	—
Oncologists		—	7	3.7
Others	10	4.4	8	4.2
No answer	4	1.8	4	2.1

Distribution of the source of information on TCIM choices among BP users (left columns) or MBP users (right columns). Numbers indicate percentages of patients. Multiple answers allowed.

**Table 5:** Pertinence of BP use among BP taking patients.

Accuracy (%of patients)	*n*	%
Products taken with correct use	49	21.5
Products taken properly but also for an incorrect usage	19	8.3
Products unproperly taken	59	25.9
Not all products were taken properly	59	25.9
Not evaluable	41	18.0

**Table 6:** Accuracy of intended use of BP.

Intended use (% of patients)	Unproperly taken for the intended use		Total	
	*n*	%	*n*	%
Boost immune system/immune response	43/134	32.1	134	58.8
Reduce/alleviate side effects of the therapy	46/88	52.3	88	38.6
Strengthen effects of the therapy	22/59	37.3	59	25.9
Reduce/alleviate pain	8/11	72.7	11	4.8
Others	8/24	33.3	24	10.5
Instead of therapy	4/4	100.0	4	1.8

Distribution of accuracy of BP-intended use among BP users (patients could indicate more than one reason).

## Data Availability

Data are available on request due to restrictions of privacy or ethical issues. The data presented in this study are not publicly available due to privacy protection of the patients that answered the questionnaire. Under specific requests by the editor or reviewers, raw data can be provided by Francesco Lozupone (e-mail: francesco.lozupone@iss.it)
